RETRACTED

# Artificial Intelligence Enterprise Management Using Deep Learning

**DOI:** 10.1155/2022/2422434

**Published:** 2022-06-17

**Authors:** Xiaofeng Liu, Li Han

**Affiliations:** School of Management, Harbin University of Commerce, Harbin, Heilongjiang, China

## Abstract

In this paper, we explore the application status of deep learning (DL) in enterprise management, with China Merchants Bank as an example, and the role of DL in bank enterprise management. We analysed the application status of AI in marketing, risk control, investment, and other fields of CMB and identified five types of problems encountered in the current practical application of AI. We proposed five countermeasures: strengthening the AI organisation system's construction, enhancing the financial data guarantee mechanism, concentrating on customer-oriented, tightly managing the danger of AI technology, and building a full AI talent system. Recent data are used to assess the impact of DL in marketing, risk management, and investment consulting. According to the data, by the end of 2019, the number of clients of CMB's two APP platforms had reached 114 million and 91.2643 million, respectively. In 2019, CMB's personal savings balance climbed by roughly 53% compared to 2016, and its personal loan amount increased by approximately 61%. These findings indicate that the use of AI improves consumer happiness and trust in businesses.

## 1. Introduction

Financial technology has ushered in a new era of transformation in the financial sector. Financial company growth using technology as a driving factor has quickly focused on financial and Internet firms. Traditional financial institutions face several issues due to the emergence of Internet financial institutions, such as shrinking profit margin and client loss. Driven by external competitive pressure and internal transformation need, banks increasingly boost the development of intelligence-related goods and services [1, 2]. In the newly announced policy, the government further states that firms are encouraged to use artificial intelligence (AI) to enterprise management and continually push computer technology to increase the digital level in the financial industry.

LeCun et al. [3] proposed the notion of DL for the first time. It is a machine learning approach based on data representation learning. The primary concept is to analyze data by mimicking human brain operations such as sight, sound, and text. The data features are automatically retrieved using the training depth model [4]. The majority of current DL research is focused on neural network approaches such as convolutional neural network (CNN), recurrent neural network (RNN), and deep belief network (DBN).  Figure 1 depicts the fundamental architecture of a neural network. Deep learning (DL) technology has recently achieved a breakthrough in the field of social digitalization. DL technology is mostly useful in the disciplines of data mining, natural language comprehension, and computer vision, exhibiting large data-driven and man-machine integration qualities. Commercial bank financial data are thought to be more suited for the DL model due to their continuity, large dimension, and temporal variability [5–7]. Meanwhile, DL's sophisticated nature and broad applicability can provide commercial banks with a plethora of novel applications in risk management and intelligent services. Exploring the scenario application of DL in the financial business may become a sharp weapon for banks to increase their intelligent service level and accomplish corner overtake [8].

RETRACTED

Although AI technology is increasingly employed in commercial banks, certain issues still need to be addressed in actual implementations. At the moment, most AI technologies in China are based on established technology from other countries. There are few in-depth studies based on instances, and the majority of them outline the function of AI unilaterally, without detailed examination. As a result, the application of AI in China Merchants Bank (CMB) is used as a case study to examine and assess the application impact of AI, highlighting existing application obstacles and proposing focused solutions.

## 2. Materials and Methods

### 2.1. Related Concepts and Analyses

An artificial neural network may be divided into three modules: the input module, the hidden module, and the output module. The input layer is responsible for receiving data. The hidden layer uses the input to execute mathematical operations to determine the connection between neurons. In the creation of neural networks, one of the most challenging aspects is selecting the number of hidden layers and the number of neurons inside each layer. In DL, the term “deep” refers to the number of hidden layers that are present. The model's prediction results are delivered by the output layer [9, 10]. At the moment, there is no universally accepted definition of DL. However, a search of relevant literature reveals that the majority of academics describe DL in terms of the four elements shown in Figure 2.

The fast expansion of the Internet and information technology has resulted in an explosion of data. The ability to process and analyze massive amounts of data in real-time presents a potential for DL development. Deep neural networks allow a computer to construct a complicated network using multilayer basic mathematical computations. The initial few levels of a multilayer neural network can learn some basic low-level features, while the final few layers gain the capacity to identify more complicated things based on the combination of simple characteristics. It can automatically learn shallow features an abstract deep multidimensional features layer by layer as the depth of the neural network and model complexity expand and improve, giving it a more complicated learning representation capacity.

RETRACTED

#### 2.1.1. Intelligent Marketing

Massive and multidimensional big data sets offer adequate circumstances for developing the DL algorithm. The development of the Graphics Processing Unit (GPU) chip compensates for the Central Processing Unit (CPU) deficiencies in parallel computing and offers computational assistance for DL algorithm research. The addition of “data + computational power” aids in advancing the DL algorithm. Major advances in computing materials, processing power, and algorithms have accelerated the development of AI technology represented by the DL algorithm, bridging the gap between theory and practice [11, 12]. AI technologies such as machine vision, voice recognition, natural language processing, and human-computer interaction are steadily moving from “cannot be used and difficult to use” to “can be used,” ushering in a new generation of AI development. In the financial sector, employing AI technology to infuse fresh life into conventional finance and expedite the transformation of science and technology has also become a hot topic. Currently, financial institutions continue to investigate the integration and deployment of AI technology and business situations, and preliminary results have been obtained. The financial sector is increasingly evolving toward an integrated and automated intelligent platform for marketing, risk management, assessment, operation, and other linkages as AI technology matures. The investigation and implementation of DL, which enables banks to cut costs, boost efficiency, and expedite scientific and technological development, are discussed.

In recent years, the conventional financial sector as a whole has confronted the conundrum of increased client attrition but reducing net profit growth. The traditional business makes it tough to earn profits and expand revenue, and scientific and technological innovation is on the horizon. Because of the innovation of the DL algorithm, many marketing methods have moved from “imagination” to “reality.” Ping and Group's One Connect uses the DL algorithm to create an integrated marketing scheme that naturally merges sophisticated technologies such as big data and AI with conventional business procedures. Deep neural networks are used to build (1) *N* facial recognition, microexpression recognition, intelligent text reading comprehension, and other technologies. Gamma Shike Glasses, Gamma Guest Screen, and Gamma Marketing Assistant are intelligent technologies developed to cover the scenes of inside and outside bank outlets, online and offline, and digital marketing [13, 14]. Bank of Shanghai trains employees to build a machine learning model in various business scenarios such as mining new customers, retaining lost old customers, and new product marketing. In the scenario of a large amount of data, given the limitations of traditional machine learning algorithms, the Bank of Shanghai explores how to build an in-depth model, improve the actual marketing effect of the model, and help the bank innovate, promote activity, retain, and generate revenue from multiple angles and dimensions.

RETRACTED

This new marketing method can solve a large part of the shortcomings of traditional offline and online marketing modes, reduce the human and material resources used in marketing, and greatly improve work efficiency. Applying AI to the marketing of bank enterprises will greatly improve banks' market competitiveness and customer satisfaction with products [15].  Figure 3 shows a comparison between traditional marketing and intelligent marketing in two aspects of customer access and marketing.

Intelligent marketing is mostly carried out in two processes, as seen in Figure 4. To correctly gather target consumers, the first step is to assess clients based on their various interests and offer relevant items to them. Following the acquisition of target customers, the second phase is to develop focused marketing programs for various customers in order to increase the connection between firms and customers and accomplish value transformation.

#### 2.1.2. Intelligent Risk Control

Intelligent risk control anticipates the risks that may emerge during the transaction by using data previously saved by consumers to determine the remedy in advance [16]. Transactions, i.e., data interchange, are always carried out in commercial banks. AI may be used to evaluate this data, identify problematic data, perform risk prediction, timely tracking, and further determine if it fits the standards of bank transactions. Furthermore, AI can warn of difficulties in bank transactions, prohibit inappropriate transactions in real-time, and significantly increase banks' risk management levels [17, 18]. For example, AI may handle the loan process when banks lend, as seen in Figure 5.

### 2.2. Application of AI in the Management of CMB

The AI recommendation system is mostly used in the CMB business management process. Other recommendation systems are available now, but the collaborative filtering algorithm is essential [19–23]. Its core concept is to examine clients and goods that may interest them. When a collaborative filtering algorithm is used in corporate management, it may be classified into two types. [22, 23] The user-based collaborative filtering algorithm (user-base) and the item-based collaborative filtering algorithm (item-base).

RETRACTED

The user base is separated into two stages. First, seek clients comparable to the target market and then gather data. Second, comparable clients are analysed to locate goods of mutual interest. If the target client does not have the product, propose it [24, 25].

When calculating the interest similarity of customers, cosine similarity can be used to replace it. If *X* customers are found interested in product {*a*, *b*, *d*} and *Y* customers are found interested in product {*a*, *c*} through data analysis, Equation (1) can be used to calculate the similarity of interest between *X* customers and *Y* customers.

(1) $$\begin{array}{c} w_{uv}=\frac{\left|N\left(u\right)\cap N\left(v\right)\right|}{\sqrt{\left|N\left(u\right)\right|\left|N\left(v\right)\right|}}. \end{array}$$

After using equation (1) to calculate the interest similarity between customers, user-based collaborative filtering algorithm can be used to recommend products that customers with high interest similarity are currently using. Interest degree of customer *u* in product *i* can be calculated by

(2) $$\begin{array}{c} p\left(u,i\right)=\sum_{v\in S\left(u,K\right)\cap N\left(i\right)}w_{uv}r_{vi}. \end{array}$$

In equation (2), *S*(*u*, *k*) represents a collection of customers with high similarity to *u* customer interest. *N*(*i*) represents collection of customers with products. Variant *w*_*uv*_ represents interest similarity of customers *u* and *v*. Variant *r*_*vi*_ represents customer *v* interest in products *i*. At this point, the interest given in the system actually represents the customer's desire to buy products.

Item-base can also be divided into two steps in the operation. First, evaluating the similarity between various products. Second, recommending similar items to customers based on similarity between products and previous purchases [26]. If most customers who like product *i* also like product *j*, then product *i* and product *j* are similar products, and equation (3) can be used to represent the similarity between product *i* and product *j*.

(3) $$\begin{array}{c} w_{ij}=\frac{\left|N\left(i\right)\cap N\left(j\right)\right|}{\sqrt{\left|N\left(i\right)\right|\left|N\left(j\right)\right|}}. \end{array}$$

In equation (3), *N*(*i*) represents collection of customers who purchased product *i*. |*N*(*i*)| represents the length of the collection of customers who have purchased product *i* and in order to make the calculation easier, the interest of *u* customers in item *I* can be represented by.

(4) $$\begin{array}{c} p_{uj}=\sum_{i\in N\left(u\right)\cap S\left(j,K\right)}w_{ji}r_{ui}. \end{array}$$

The advantages and disadvantages of the two algorithms are compared in Figure 6.

RETRACTED

Figure 7 shows the business flow of the recommending system.

### 2.3. Analyses on the Role of AI in Enterprise Management of CMB

The role of AI in CMB enterprise management can be divided into three aspects as shown in Figure 8.

#### 2.3.1. AI Algorithm to Promote Intelligent Marketing

In order to get target consumers via many channels, assess customers, adapt marketing programs for individual customers, and propose items that customers may be interested in, CMB employs artificial intelligence (AI) in its marketing strategy. These are the three components of CMB's marketing characteristics that are worth noting: first and foremost, it collects the targeted clients via a variety of channels. For example, when CMB conducts business, it will very definitely rely on the two CMB and Palm Life Apps, which serve as the company's primary Internet access channels. Second, it creates multichannel Internet access channels with the use of the WeChat public number platform, which is powered by Tencent. In addition, CMB employs collaborative marketing, brand advertising marketing, and We-media fans marketing, all of which contribute to a significant rise in the number of clients. For the third time, a differentiated marketing approach for distinct clients is implemented. Customers are divided into groups by their ages, according to the bank's classification system. When hotspots and headlines are used together, the bank may strengthen its brand recognition across all age groups while also increasing consumers' viscosity and confidence in corporate entities [27, 28].

#### 2.3.2. Assistance of AI to Intelligent Risk Control

When CMB performs risk control, it suggests a new system—the “Libra System,” which is based on an artificial intelligence algorithm. When clients perform transactions, the Libra System may collect multidimensional data such as the time, the amount, and the payee. It is vital to analyze the data gathered above via a risk control algorithm to make it easier for consumers to estimate their own risks. According to the findings of the data analysis, customer groups with varying degrees of risk must be recognized in various ways to analyze possible safety threats throughout the transaction process [29].

RETRACTED

For the time being, CMB relies mostly on the common debt risk identification and postloan automated monitoring systems to forecast and avoid hazards associated with common debt obligations. The following is the primary procedure for determining the danger of shared debt. In order to integrate the various data of customers, including transaction data and external information, generate the asset perspective of customers, understand the current property status of customers, evaluate whether the user can pay off the debt within the specified time frame, and finally make the decision whether to lend to the user, artificial intelligence technology is used in this process. After a bank has loaned money to a client, the automated monitoring system might continue to watch the consumer's progress. When clients have credit difficulties, CMB will implement a number of measures to lessen the likelihood of default. Aside from this, CMB links retail and business customers, analyses and combines the data of various kinds of consumers, and acquires a huge data collection in order to lower the risk of default associated with the transaction.

CMB's retail credit intelligent approval robot will be formally released on April 28, 2020. AI is completely applied to the loan approval link, significantly reducing the approval link's consumption of human and material resources and enhancing job efficiency. The robot can examine clients prior to formal loans and synthesize various approval opinions in the database to provide approval opinions for CMB applicants in a matter of seconds. So far, the intelligent approval robot has saved the bank 21% of its approval time while efficiently spotting potential dangers. The number of retail loans evaluated has surpassed 300,000, and the total amount sanctioned has surpassed 260 billion yuan.

#### 2.3.3. AI Algorithms Lead Intelligent Investment Consultants

As one of the first bank companies in China to use intelligent investment, CMB released the Capricorn Intelligent Investment product at the end of 2016, which offers a new way for growing intelligent investment and financing of domestic banks [30]. Capricorn Intelligence Investment is built using contemporary portfolio theory as its theoretical foundation and AI technologies such as computer learning algorithms as its technical backing. It combines CMB's many years of operating and management knowledge to provide an intelligent fund investing system for the majority of the world's investors. The “Capricorn Intelligent Investment” system is China's first intelligent investment system. Its primary work procedure is as follows. The bank funds are categorised using the recommended system model. In the face of diverse investors, risk tolerance, capital status, investment time limit, and other factors should be thoroughly evaluated, and funds in the current market should be screened to propose the most appropriate funds for investors, and customers should be regularly watched. Customers should be presented with important information on a continuous basis. The most significant benefit of this system is its ability to employ AI to give individualised suggestions to clients in order to suit their demands in all areas.

RETRACTED

After CMB implements the Capricorn Intelligent Investment System, it will be able to consider both “Golden Sunflower” and “Long Tail” clients, saving time on prospective mining customers [31]. According to the relevant statistics from the CMB Annual Report in 2018, the total acquisition amount of Capricorn Investment System has surpassed 12 billion yuan. Simultaneously, “Capricorn Intelligent Investing” primarily intends to apply AI to investment. Therefore, future development of “Capricorn Intelligent Investment” will concentrate on intelligent interaction [32, 33].

## 3. Results

### 3.1. Effectiveness Analyses of Intelligent Marketing

CMB employs AI to precisely determine the business model of target clients, which significantly enhances the user activity of the CMB APP and Palm Life APP. From 2016 to 2019, the number of users of the two software packages was statistically examined. The precise data are shown in Figures 9 and 10.

According to Figure 8, the number of CMB APP and Palm Life APP users increases. By 2019, CMB software users will have surpassed 114 million. CMB APP has the most users compared to the eight major joint-stock banks, and the frequency with which users utilize CMB APP is rather high, with an average of roughly 12 logins each month. In 2019, the total number of APP users was around three times 2016, reaching 91.26 million homes.

Furthermore, the marketing technique of gathering user information and tailoring suggestions for users increases user viscosity for firms. As a result, CMB's personal deposit and loan balances are gradually expanding. The particular values are shown in Figure 11.

As illustrated in Figure 11, CMB's deposit and loan balances have increased steadily since 2016. Compared to the balance in 2016, the individual deposit balance of CMB in 2019 has climbed by about 53%, and the individual loan amount has increased by nearly 61% to 24,753. Individual loan balances are expanding faster than individual deposit balances. According to the evidence shown above, the introduction of AI significantly improves customer pleasure and confidence in CMB.

### 3.2. Effectiveness Analysis of Intelligent Risk Control

It is critical to use AI in risk management in CMB. Three typical instances are as follows:

1. Since the “scale system” was established in early 2016, almost $3 billion in transactions have been safeguarded. When a transaction risk arises, the system will reply, with a response time of 30 milliseconds. The system can make judgments in advance even if the user has not yet noticed the danger, thereby protecting the user's financial security. In 2019, the system prevented 80,000 telephone fraud transactions, safeguarding over CNY 1.8 billion in customer payments.
2. In terms of nonperforming loan percentages, CMB has progressively decreased since 2016. CMB's nonperforming loan ratio was just 1.13% in the third quarter of 2020, down 0.03% from the end of 2019, the provisional loan ratio declined by 0.18%, and the coverage of provisional nonperforming loans decreased by 2.02%.  Figure 12 depicts information.
3. As shown in Figure 12, the percentage of nonperforming loans for CMB in 2016 was as high as 1.87%, and the nonperforming loan rate has been reduced in subsequent years. The explanation for this may be found in the fact that, since 2017, CMB has started to deploy intelligent risk control technology to enterprise risk management, suggesting that AI has a positive influence on avoiding nonperforming loans. CMB's company continued to grow in the face of the pandemic in 2020. In this scenario, CMB's nonperforming loan rate did not increase but gradually fell, indicating that the external environment will not disrupt the bank's overall risk management capabilities if AI is used.
4. Since 2016, the loan migration ratio of CMB has begun to show a steady downward trend. With the help of intelligent risk control systems, the normal loan migration rate in 2019 has fallen to half of that in 2016, indicating that CMB has a strong loan collection capacity for initially expected loans. For suspicious loans, except for 2019, the migration rate of suspicious loans is declining, and it dropped to 19.9% in 2018. It shows that CMB can timely and effectively control the risk of such loans to prevent more nonperforming loans.  Figure 13 shows specific data.

RETRACTED

### 3.3. Effectiveness Analysis of “Capricorn Intelligent Investment”

Since implementing the “Capricorn Intelligent Investment,” sales of CMB mobile phone financial products have surged significantly.  Figure 14 depicts the particular sales share of mobile banking financial products from 2017 to 2019.

Figure 14 shows that CMB's mobile phone financial goods sales exceeded 6 trillion yuan in 2018, with overall CMB product sales exceeding 10 trillion yuan this year. In 2018, mobile financial products account for more than half of the total sales of financial products, and this figure increased in 2019. When CMB provides financial goods, mobile Internet banking is the preferred method. In this scenario, “Capricorn Intelligent Investment” steadily demonstrates its value to the business.

Furthermore, as the first domestic smart investment product, “Capricorn Intelligent Investment” has collected sales of 12.233 billion yuan, indicating that it can achieve consistent sales development without creating huge swings. This trait allows it to thrive during a capital market slump. CMB allows consumers to earn significant returns and regularly updates and enhances the “Capricorn Intelligent Investment” system to increase user satisfaction with intelligent technologies.

### 3.4. Opportunities for DL Development

The DL algorithm's large-scale implementation is still a long way off. It remains focused on research in the medium term, with a tiny amount of realization serving as an auxiliary function. However, the potential of DL to encourage the growth of the banking sector should not be overlooked nor should its beneficial function be understated.

#### 3.4.1. More Exceptional Data Value

With the advent of huge external information in the age of big data and the growth of internal business, staff, and system platforms, the issue of data island becomes more significant. Furthermore, institutions are becoming more cognizant of the significance of data. The federated learning method eliminates data obstacles imposed by security and privacy concerns. The combination of federated learning and DL algorithms can incorporate multidimensional data mining and analysis characteristics, avoiding waste from direct storage and increasing the value of big financial data.

#### 3.4.2. Improved Service Intelligence

The advancement of DL makes computers more human-like and capable of providing consumers with humanized and tailored services in batches, significantly influencing the banking sector at the top end of the service value chain. It will usher in a new wave of changes to financial products, service channels, service methods, and risk management, fundamentally altering the financial industry's current pattern and making financial services (banking, insurance, financial management, lending, and investment) more personalized and intelligent.

#### 3.4.3. Increased Risk-Management Capabilities

Because the financial system is always under assault from various sources, the standard artificial risk control model cannot cope with hazards when dealing with complex data such as risk management and transactions. With the introduction of DL technology, the model can automatically learn and forecast hazards, which may significantly cut human costs, increase financial risk management and business processing capacity, and improve the overall security and stability of the financial system.

RETRACTED

AI technology is continually improving as DL technology advances. Commercial banks should collaborate with all industry stakeholders to continuously improve top-level design, strengthen core technology research, collaborate to improve the data ecosystem, promote the popularization and development of AI technology in the banking industry, innovate service methods and processes, improve the overall banking industry's resource allocation efficiency, and respond to customers' and society's needs in a more advanced, flexible, and efficient manner.

## 4. Conclusions

As the backbone of the national economy, the banking sector has also ushered in a historic breakthrough. Traditional marketing management techniques have failed to adapt to today's diverse societal requirements. To strengthen their competitiveness, banks must use clever management techniques. The research investigates the usage of AI in CMB's enterprise management using the case analysis approach. Starting with the idea of a recommendation system, the article explains the current state of AI technology in CMB, examines its application impact using recent data, and offers solutions to challenges found in practice. However, due to AI technology's fast advancement, it will be impossible for the article to cover all conceivable future AI technologies. There is still a gap compared to expert research, and there is a need for ongoing learning improvement.

## Figures and Tables

**Figure 1:** Basic principle and architecture of the neural network.

**Figure 2:** Definition of DL from different angles.

**Figure 3:** Comparison between traditional marketing and intelligent marketing.

**Figure 4:** Steps of intelligent marketing.

**Figure 5:** The role of AI in loan approval process.

**Figure 6:** Comparison of the advantages and disadvantages of user-base algorithm and item-base algorithm.

**Figure 7:** Flow of the recommending system.

**Figure 8:** The role of AI algorithms in commercial banks.

**Figure 9:** Individual deposit and loan balance of CMB.

**Figure 10:** Users of joint stock bank mobile banking in 2019.

**Figure 11:** Individual deposit and loan balance of CMB.

**Figure 12:** Nonperforming loan ratio of CMB, 2016–2020.

**Figure 13:** Loan migration rate indicators of CMB.

**Figure 14:** Proportion of financial sales of CMB on mobile banking.

## Data Availability

The experimental data used to support the findings of this study are available from the corresponding author upon request.
